The article "Epstein–Barr virus-encoded microRNA BART1 induces tumour metastasis by regulating PTEN-dependent pathways in nasopharyngeal carcinoma" was retracted in 2025. Reasons: contaminated cell lines or tissues; duplicated images; overlap with earlier publications; unreliable data.

# Epstein–Barr virus-encoded microRNA BART1 induces tumour metastasis by regulating PTEN-dependent pathways in nasopharyngeal carcinoma

**DOI:** 10.1038/ncomms8353

**Published:** 2015-07-02

**Authors:** Longmei Cai, Yanfen Ye, Qiang Jiang, Yuxiang Chen, Xiaoming Lyu, Jinbang Li, Shuang Wang, Tengfei Liu, Hongbing Cai, Kaitai Yao, Ji-Liang Li, Xin Li

**Affiliations:** 1 Cancer Research Institute, Southern Medical University, Guangzhou 510515, China; 2 Radiation Department, The First Affiliated Hospital, Wannan Medical College, Wuhu 241001, China; 3 Department of Pathology, Basic Medical College, Southern Medical University, Guangzhou 510515, China; 4 School of Traditional Chinese Medicine, Southern Medical University, Guangzhou 510515, China; 5 School of Biotechnology, Southern Medical University, Guangzhou 510515, China; 6 Molecular Oncology Laboratories, Department of Oncology, Weatherall Institute of Molecular Medicine, University of Oxford, John Radcliffe Hospital, Oxford OX3 9DS, UK

## Abstract

Epstein–Barr virus (EBV), aetiologically linked to nasopharyngeal carcinoma (NPC), is the first human virus found to encode many miRNAs. However, how these viral miRNAs precisely regulate the tumour metastasis in NPC remains obscure. Here we report that EBV-miR-BART1 is highly expressed in NPC and closely associated with pathological and advanced clinical stages of NPC. Alteration of EBV-miR-BART1 expression results in an increase in migration and invasion of NPC cells *in vitro* and causes tumour metastasis *in vivo*. Mechanistically, EBV-miR-BART1 directly targets the cellular tumour suppressor PTEN. Reduction of PTEN dosage by EBV-miR-BART1 activates PTEN-dependent pathways including PI3K-Akt, FAK-p130^Cas^ and Shc-MAPK/ERK1/2 signalling, drives EMT, and consequently increases migration, invasion and metastasis of NPC cells. Reconstitution of PTEN rescues all phenotypes generated by EBV-miR-BART1, highlighting the role of PTEN in EBV-miR-BART-driven metastasis in NPC. Our findings provide new insights into the metastasis of NPC regulated by EBV and advocate for developing clinical intervention strategies against NPC.

## Abstract (web summary)

Epstein–Barr virus is associated with nasopharyngeal carcinoma and previous studies have focused on the role of viral proteins in tumour pathology. Here, the authors show that a viral miRNA targets the host protein PTEN and has a critical role in the late stage of nasopharyngeal carcinoma by driving tumour metastasis.

Nasopharyngeal carcinoma (NPC) represents a serious health problem in Southern China and Southeast Asia and has a high metastatic potential. Most patients with the disease are diagnosed only when the tumour has reached an advanced stage (stages III and IV)^1^. Interactions among environmental carcinogens, genetic alternations and viral infections are believed to play a major role in the pathogenesis of NPC^2^. However, the molecular mechanisms for the metastases of NPC remain obscure.

The article "Epstein–Barr virus-encoded microRNA BART1 induces tumour metastasis by regulating PTEN-dependent pathways in nasopharyngeal carcinoma" was retracted in 2025. Reasons: contaminated cell lines or tissues; duplicated images; overlap with earlier publications; unreliable data.

The Epstein–Barr virus (EBV), latently infected >90% of the global population, is aetiologically linked to several human lymphocytic and epithelial malignancies including Burkitt's lymphoma, Hodgkin's disease, post-transplant lymphoma, gastric cancer (GC) and NPC^3^. To date, most studies have focused on EBV-encoded proteins such as the latent nuclear antigen EBNA1 (ref. 4) and the latent membrane proteins LMP1, LMP2A and LMP2B, which have the abilities to transform cells, to alter cellular gene expression and to increase the growth, survival and invasion of transformed cells^4^,^5^. However, EBV-associated tumours usually express a restricted repertoire of viral proteins in a histological specific fashion^6^, suggesting that the pathogenesis and progression of these tumours are not only regulated by viral proteins but also by other important factors such as EBV-encoded microRNAs (EBV-miRs).

MicroRNAs (miRNAs), a class of 17–23 nucleotide non-coding RNAs, are capable of inhibiting the expression of multiple target genes by forming imperfect complementary duplexes with their target mRNAs in the 3′-untranslated region (3′-UTR), leading to mRNA degradation or translational inhibition^7^, and participate in diverse biological processes including tumorigenesis and metastasis^8^. EBV is the first human virus found to encode miRNAs^9^. To date, a total of 25 EBV-miR precursors containing 48 mature miRNAs have been identified within two regions of the EBV genome. The BamHI fragment H rightward reading frame 1 (BHRF1) gene encodes 3 miRNA precursors (that is, EBV-miR-BHRF1 1–3) generating four mature miRNAs, while the BamHI fragment A rightward transcript (BART) region contains 22 miRNA precursors (that is, EBV-miR-BART1-22) producing 44 mature miRNAs^10^,^11^,^12^. The abundance of individual miRNAs within cell lines and tumour tissues varies widely and appears to be cell-type and tumour-type specific. The expression of EBV-miR-BHRF1 was highly restricted to lytic and latency III-infected cell lines such as B lymphoma cells, whereas EBV BART miRNAs were detected in all types of EBV-associated latency^10^,^13^,^14^,^15^,^16^,^17^,^18^,^19^,^20^,^21^. Interestingly, the expression of BART miRNAs was shown to be relative low in EBV-infected B lymphocytes but extremely high in infected epithelial tissues, suggesting a pathogenic role in the development of epithelial malignancies^15^,^17^,^21^,^22^,^23^.

The article "Epstein–Barr virus-encoded microRNA BART1 induces tumour metastasis by regulating PTEN-dependent pathways in nasopharyngeal carcinoma" was retracted in 2025. Reasons: contaminated cell lines or tissues; duplicated images; overlap with earlier publications; unreliable data.

Many EBV BART miRNAs were found highly expressed in NPC and GC^22^,^24^,^25^, contributing to viral latency^23^,^26^,^27^, host cell survival^25^,^27^ and immune escape^28^. However, their functions in tumorigenesis and tumour progression of NPC remain elusive. We are interested in the viral and cellular miRNAs in the tumour biology and clinical significance in NPC^29^,^30^. In this study, we report that EBV-miR-BART1 is highly expressed in NPC and closely associated with pathoclinical features of NPC. Alterations of the expression of EBV-miR-BART1 demonstrated that it induces the migration and invasion of NPC cells *in vitro* and the tumour metastasis *in vivo.* The underlying molecular mechanisms by which BART1 causes tumour metastasis are revealed to directly target the major tumour suppressor, phosphatase and tensin homologue (PTEN) and consequently to activate PTEN-dependent pathways and induce epithelial–mesenchymal transition (EMT). Our findings provide new insights into the metastasis of NPC regulated by EBV and advocate for developing clinical intervention strategies for NPC.

## Results

### EBV-miR-BART1 is associated with pathoclinical features

We performed miRNA expression profile microarray analysis of 20 NPC versus 20 non-cancerous nasopharyngeal (NP) tissues (Supplementary Table 1) and identified 69 miRNAs that were differentially expressed between NPC and NP samples (Fig. 1a). Of them, 24 miRNAs were upregulated and 45 miRNAs were downregulated in NPC specimens. Intriguingly, among all upregulated miRNAs, 62.5% (15/24) were EBV BART miRNAs, while only 29.2% (7/24) were human cellular miRNAs (Supplementary Table 2). In contrast, all downregulated miRNAs were host derived, of which a large proportion (55.6%, 25/45) were tumour suppressive miRNAs such as the let-7 family (hsa-let-7c, d, g and i)^31^, miR-34 family (miR-34c and d)^32^, miR-29 family (miR-29a, b and c)^32^, miR-30 family (miR-30a-5p, 30a-3p, b, d and e)^33^, miR-26 family (miR-26a and b)^34^, miR-143/145 cluster^35^, miR-16 (ref. 36), miR-31 (ref. 37), miR-101 (ref. 38), miR-146a^39^, miR-150 (ref. 40), miR-152 (ref. 41) and miR-195 (ref. 42). Notably, BART1, BART7, BART3, BART10, BART8, BART9 and BART5 were in the top seven and clustered together, suggesting that EBV BART miRNAs may play a critical role in NPC.

To investigate if the EBV-miR-BART1 expression is associated with pathoclinical features of NPC, we determined the expression of EBV-miR-BART1 in another cohort of 82 NPC samples that contain the TNM-stage information (Supplementary Table 3). The expression of either BART1-5p (3.8-fold) or BART1-3p (2.9-fold) was dramatically increased in N2–3 stages as compared with N0–1 stages (Fig. 1b). Similarly, a substantial higher level of BART1-5p (3.4-fold) or BART1-3p (3.0-fold) was observed in advanced clinical stage III–IV than in early clinical stage I–II (Fig. 1c). Thus, the results suggest that EBV-miR-BART1 might contribute to the metastasis of NPC.

The article "Epstein–Barr virus-encoded microRNA BART1 induces tumour metastasis by regulating PTEN-dependent pathways in nasopharyngeal carcinoma" was retracted in 2025. Reasons: contaminated cell lines or tissues; duplicated images; overlap with earlier publications; unreliable data.

### EBV-miR-BART1 impels NPC metastasis *in vitro* and *in vivo*

We upregulated the expression of BART1 in two EBV-negative NPC cell lines (CNE1 and 5-8F) by lentivirus-mediated transduction (Supplementary Fig. 1). Transwell migration assays (Fig. 2a) and wound-healing assays (Supplementary Fig 2) demonstrated that upregulation of BART1 dramatically increased the cell migration of either CNE1-BART1 or 5-8F-BART1 compared with relative mock control. Boyden chamber invasion assays (Fig. 2b) revealed that the upregulation of BART1 significantly increased the cell invasion of both CNE1-BART1 and 5-8F-BART1 compared with the relative control. To verify the results, we downregulated the expression of BART1 in CNE1-BART1 and 5-8F-BART1 by transfection of BART1-inhibitory oligonucleotides (Supplementary Fig. 3). Consistent with the upregulation results, downregulation of BART1 by either in-b1-5p or in-b1-3p dramatically decreased the migration (Fig. 2c) and invasion (Fig. 2d) of either CNE1-BART1 or 5-8F-BART1 cells compared with the relative in-NC control. An additive effect on cell migration or invasion was observed when combined the two BART1 inhibitors (Fig. 2c,d). Together these results suggest that EBV-miR-BART1 propels the migration and invasion of NPC cells *in vitro*.

We xenografted 5-8F-BART1 cells into nude mice. Upregulation of BART1 significantly increased the tumour growth of 5-8F-BART1 compared with the 5-8F-mock control (Fig. 2e,f). Transplantation of 5-8F cells underneath the liver envelope^43^,^44^ demonstrated that the upregulation of BART1 promoted the tumour metastasis of 5-8F-BART1 compared with the 5-8F-mock control (Fig. 2g). Three weeks after the transplantation, 86% of mice (6/7) in the 5-8F-BART1 group showed both liver and lymph node metastases compared with 14% of mice (1/7) in the 5-8F-mock group (Chi-square test *P*<0.05); 43% of mice (3/7) in the 5-8F-BART1 group displayed lung metastasis compared with 14% of mice (1/7) in the control group (Fig. 2h). In the metastasized lymph nodes, 45 tumour nodules in the 5-8F-BART1 tumours were observed compared with five nodules in the control tumours (6.43±2.13 versus 0.71±0.71, Student's *t* test *P*<0.05; see Fig. 2h). Re-examination of EBV-miR-BART1 expression in liver-metastasized tumours by quantitative reverse transcription PCR (qRT–PCR) demonstrated that the metastasized tumour cells stably expressed BART1-5p and BART1-3p at the levels close to that of NPC clinical samples (Supplementary Fig. 4). Thus, the results indicate that EBV-miR-BART1 impels the growth and metastasis of NPC cells *in vivo.*

The article "Epstein–Barr virus-encoded microRNA BART1 induces tumour metastasis by regulating PTEN-dependent pathways in nasopharyngeal carcinoma" was retracted in 2025. Reasons: contaminated cell lines or tissues; duplicated images; overlap with earlier publications; unreliable data.

### EBV-miR-BART1 directly targets cellular PTEN in NPC cells

We investigated BART1-targeted genes that are associated with tumour metastasis by developing an integrated strategy (Fig. 3a). RNA-deep sequencing analysis of the gene expression profiling of CNE1-BART1 cells versus CNE1-mock cells identified 995 downregulated genes, from which many metastasis-associated candidates can be retrieved (Supplementary Table 4 and Supplementary Fig. 5). Pathway enrichment analysis for these downregulated genes revealed that BART1 regulated many important signalling pathways such as p53 signalling pathway, pathway in cancer, MAPK pathway, regulation of actin cytoskeleton, Jak-STAT signalling pathway and focal adhesion pathway. At least 10 genes were significantly altered in each of these pathways by BART1. PTEN was identified as one of the top genes regulated by BART1 and involved in five tumour metastasis- or cell invasion-associated pathways.

Bioinformatics analysis showed that PTEN 3′-UTR region contains two sites complementary with the seed sequences of BART1-5p and BART1-3p from the nucleotide position 425 and 921, respectively (Fig. 3b). To clarify if PTEN is a direct cellular target for BART1, we performed luciferase reporter assays by co-transfection of a wild-type (wt) or mutant (mut 1 or mut 2) PTEN 3′-UTR-containing luciferase reporter vector with a BART1 mimic. The luciferase activity of the wt PTEN 3′-UTR but not the mutant 3′-UTR (either mut 1 or mut 2) was significantly reduced by b1-5p mimic alone or b1-3p mimic alone but not by the control mimic (NC). The combination of b1-5p with b1-3p produced an additive effect on the luciferase activity (Fig. 3c).

The effects of EBV-miR-BART1 on PTEN mRNA and protein expression were examined in NPC cell lines, xenografted tumours and clinical samples. Upregulation of BART1 significantly reduced the expression of PTEN in both CNE1-BART1 and 5-8F-BART1 cell lines compared with the relative control as revealed by western blotting and immunofluorescent (IF) staining (Fig. 3d, upper panels). Immunohistochemical (IHC) staining on tumour sections of xenografts and metastasized organs demonstrated that the upregulation of BART1 significantly reduced the expression of PTEN in 5-8F-BART1 tumours compared with the 5-8F-control tumours (Fig. 3d, lower panels). Detection of the PTEN mRNA by qRT–PCR revealed that the expression of PTEN in clinical tumour samples was significantly decreased in N2–3 stages as compared with either N0–1 stages (0.1673±0.0295 versus 0.3927±0.0435, *P*<0.0001) or NP (0.1673±0.0295 versus 1.2100±0.1247, *P*<0.0001; Fig. 3e, left panel). Similarly, the expression of PTEN was significantly lower in advanced clinical stages III–IV than in either early clinical stages I–II (0.1683±0.0210 versus 0.4088±0.0331, *P*<0.0001) or NP (0.1683±0.0210 versus 1.2100±0.1247, *P*<0.0001; Fig. 3e, right panel). Strikingly, the expression of PTEN in NPC was highly inversely correlated with the expression of either BART1-5p (*r*=−0.5205, *P*<0.0001; Fig. 3f, right panel) or BART1-3p (*r*=−0.3687, *P*=0.0007; Fig. 3f, left panel). Taken together, these data indicate that PTEN is a direct cellular target of EBV-miR-BART1 in NPC.

The article "Epstein–Barr virus-encoded microRNA BART1 induces tumour metastasis by regulating PTEN-dependent pathways in nasopharyngeal carcinoma" was retracted in 2025. Reasons: contaminated cell lines or tissues; duplicated images; overlap with earlier publications; unreliable data.

### EBV-miR-BART1 activates PTEN-dependent signalling pathways

We examined the expression alterations of key components of PTEN-dependent pathways in NPC. Western blotting showed that the upregulation of BART1 significantly reduced the protein level of PTEN but increased the phosphorylation level of p-Akt, p-FAK, p130^Cas^, p-Shc or p-ERK1/2 in either CNE1-BART1 or 5-8F-BART1 cells when compared with the relative control (Fig. 4a). On the contrary, downregulation of BART1 by in-b1-5p alone, in-b1-3p alone or both inhibitors increased the PTEN level but decreased the phosphorylation of p-Akt, p-FAK, p130^Cas^, p-Shc or p-ERK1/2 in both CNE1-BART1 and 5-8F-BART1 cells (Fig. 4b). IHC staining on tumour sections of xenografts and metastasized organs demonstrated that the upregulation of BART1 significantly reduced the expression of PTEN (see Fig. 3d) but clearly increased the phosphorylation levels of p-Akt, p130^Cas^, p-Shc and p-ERK1/2 in 5-8F-BART1 tumours compared with the 5-8F-mock tumours (Fig. 4c). Collectively, these results indicate that EBV-miR-BART1 activates PTEN-dependent signalling pathways by decreased PTEN in NPC.

### EBV-miR-BART1 compels EMT

We investigated the expression of E-cadherin, N-cadherin and vimentin, as well as the rearrangement of actin cytoskeleton, a characteristic event of EMT. Western blotting demonstrated that the upregulation of BART1 strikingly decreased the expression of E-cadherin but increased the expressions of N-cadherin and vimentin in both CNE1-BART1 and 5-8F-BART1 cells compared with the relative control cells (Fig. 5a). In agreement with the upregulation results, downregulation of BART1 by in-b1-5p alone, in-b1-3p alone or both inhibitors increased the E-cadherin expression but decreased the expression of N-cadherin and vimentin in both CNE1-BART1 and 5-8F-BART1 cells as compared with the in-NC control (Fig. 5b). IHC staining on tumour sections of xenografts and metastasized organs demonstrated that the upregulation of BART1 overtly reduced the E-cadherin expression but increased the expression of vimentin in 5-8F-BART1 tumours compared with the 5-8F-mock control tumours (Fig. 5c).

The article "Epstein–Barr virus-encoded microRNA BART1 induces tumour metastasis by regulating PTEN-dependent pathways in nasopharyngeal carcinoma" was retracted in 2025. Reasons: contaminated cell lines or tissues; duplicated images; overlap with earlier publications; unreliable data.

We then performed IF staining for F-actin with Rhodamine-phalloidin. Confocal microscopy examinations showed that the upregulation of BART1 modestly increased the expression density of F-actin and triggered actin cytoskeleton rearrangement in both CNE1-BART1 and 6-8F-BART1 cells as compared with that of relative mock control cells. The organization of the actin bundles and associated proteins underneath the cell membranes (that is, cortical actin cytoskeleton) was clearly observed in either CNE1-mock or 5-8F-mock cells. In sharply contrast, dynamic structures of actin filaments and associated proteins (that is, actin stress fibre) throughout the cells, characteristic of migrating mesenchymal cells^45^, were explicitly visualized in both CNE1-BART1 and 5-8F-BART1 cells (Fig. 5d). Taken together, the results suggest that EBV-miR-BART1 promotes cell motility and invasiveness by driving EMT and increasing actin stress fibres in NPC cells.

### Restored PTEN rescues the phenotypes produced by BART1

We transfected the PTEN expression vector into CNE1-BART1 and 5-8F-BART1 cells. Restitution of PTEN expression (Supplementary Fig 6) significantly reduced the migration (Fig. 6a) and invasion (Fig. 6b) of both CNE1-BART1 and 5-8F-BART1 cells compared with the relative PTEN-negative plasmid control (NC). Detection of the key components of PTEN-dependent pathways by western blotting demonstrated that the restoration of PTEN protein decreased phosphorylation levels of p-Akt, p-FAK, p130^Cas^, p-Shc and p-ERK1/2 in both CNE1-BART1 and 5-8F-BART1 cells compared with the relative NC control (Fig. 6c). In addition, reinstallation of PTEN markedly increased the expression of E-cadherin but decreased protein levels of N-cadherin and vimentin in both CNE1-BART1 and 5-8F-BART1 cells compared with the relative NC control (Fig. 6d). Clearly, the reconstitution of PTEN emulated the results obtained from the downregulation of EBV-miR-BART1 by in-b1 inhibitors (see Fig. 2c,d, Fig. 4b and Fig. 5b).

### Reproducibility of the phenotypes in EBV-positive NPC cells

We quantified the expression of EBV-miR-BART1 in three EBV-positive NPC cell lines (that is, C666-1-EBV, HONE1-EBV and HK1-EBV) by qRT–PCR. The expression levels of both BART1-5p and BART1-3p were found comparable among three EBV-positive cell lines although lower in the cell lines than in NPC clinical samples (Supplementary Fig. 7a). We used HONE1-EBV cell line as a representative to validate the function of BART1 in NPC metastasis and underlying molecular mechanisms.

The article "Epstein–Barr virus-encoded microRNA BART1 induces tumour metastasis by regulating PTEN-dependent pathways in nasopharyngeal carcinoma" was retracted in 2025. Reasons: contaminated cell lines or tissues; duplicated images; overlap with earlier publications; unreliable data.

Transwell migration and Boyden chamber invasion assays demonstrated that the downregulation of endogenous BART1 by either in-b1-5p or in-b1-3b (Supplementary Fig. 7b) significantly decreased the migration (Fig. 7a) and invasion (Fig. 7b) of HONE1-EBV cells compared with the in-NC control. An additive effect was obtained when combined the two BART1 inhibitors (see Fig. 7a,b). Examination of the key components of PTEN-dependent pathways by western blotting showed that the downregulation of endogenous BART1 increased PTEN expression but decreased the phosphorylation of p-Akt, p-FAK and p-ERK1/2 in HONE1-EBV-positive cells compared with the in-NC control (Fig. 7c). In agreement with the results obtained from EBV-negative NPC cell lines (see Fig. 5b), downregulation of endogenous BART1 increased E-cadherin expression but decreased the expression of N-cadherin and vimentin in HONE1-EBV cells compared with the in-NC control (see Fig. 7c). Thus, the results from the EBV-positive cell line substantiate that EBV-miR-BART1 promotes cell motility and invasiveness by activating PTEN-dependent signalling pathway and driving EMT.

## Discussion

In this study, we have demonstrated that EBV-miR-BARTs are highly upregulated while cellular miRNAs are largely downregulated in NPC specimens. EBV-miR-BART1, 7, 3, 10, 8, 9, 5, 6, 2, 14 and 16 were all upregulated (Supplementary Table 2), reminiscent of the pattern of abundance of individual BART miRNAs in C666-1-EBV-positive cell line, C15 xenograft tumour and clinical samples of NPC^10^,^15^,^16^,^20^,^24^,^46^, highlighting the association of latent EBV infection with NPC and the importance of EBV BART miRNAs in NPC. Surprisingly, more than half (55.6%) of the downregulated miRNAs are tumour suppressor miRNAs, including the let-7 family, miR-34 family, miR-29 family, miR-30 family, miR-26 family, miR-143/145 cluster, miR-16, miR-31, miR-101, miR-146a, miR-150, miR-152 and miR-195, suggesting that effects of EBV infection on NPC may be partially through regulating the abundance of cellular tumour suppressive miRNAs. Consistent with our findings, EBV-infected AGS cells were shown to decrease the overall abundance of human miRNAs with specific downregulation of three types of tumour suppressive miRNAs, let-7 family, miR-200 family and miR-143 (refs 5, 16).

Several of these upregulated EBV BART miRNAs have been partially defined in epithelial carcinomas such as BART5 that inhibited cell apoptosis through targeting PUMA^25^, BART3* that promoted cellular growth by targeting DICE1 (ref. 47), BART5, 1-5p, 16 and 17-5p that have been linked to viral latency by targeting LMP1 (refs 23, 48), BART9 that increased tumour metastasis by targeting E-cadherin^49^, and BART7-3p that promoted tumour metastasis by regulation of the PTEN-PI3K/Akt-EMT pathway^50^. Here we demonstrated that EBV-miR-BART1 is closely associated with pathological and clinical stages, suggesting that BART1 may contribute to NPC metastasis, underscoring the clinical significance. To test this hypothesis, we modulated the expression of BART1 in both EBV-negative and EBV-positive NPC cells and revealed that BART1 significantly propels the migration and invasion of NPC cells *in vitro* and the tumour metastasis *in vivo* animal models. Thus, our findings shed new lights on the association of EBV BART miRNAs with NPC metastasis.

The article "Epstein–Barr virus-encoded microRNA BART1 induces tumour metastasis by regulating PTEN-dependent pathways in nasopharyngeal carcinoma" was retracted in 2025. Reasons: contaminated cell lines or tissues; duplicated images; overlap with earlier publications; unreliable data.

To explore underlying mechanisms of EBV-miR-BART1 in NPC invasion and metastasis, we exploited the integrated strategy consisting of RNA-deep sequencing, literature retrieval and pathway enrichment analysis, bioinformatics prediction, luciferase reporter assay and expression validation of targeted gene in cell lines, xenograft tumours and clinical samples to investigate targeted genes and related signalling pathways. We have identified 995 downregulated genes and many important pathways regulated by BART1. We found that PTEN is the major cellular target of BART1 in NPC. PTEN, one of the most frequently mutated and deleted tumour suppressor in the multitude of tumour types^51^, has frequently been reported downregulated in NPC^52^,^53^ while the mutation or deletion of PTEN has rarely been detected in oral squamous cell carcinoma^54^, suggesting other mechanisms in NPC are likely responsible for the downregulation of PTEN. Consistently, we found that the expression of PTEN is extremely lower (4.4-fold) in NPC than that of NP and highly inversely correlated with the expression of BART1-5p or BART1-3p in NPC. More strikingly, the expression PTEN is decreased by 2.4-fold in advanced clinical stages III–IV compared with that of early clinical stages I–II, concomitant with the higher expression of BART1 (3.4-fold for BART1-5p, 3.0-fold for BART1-3p) in advanced stages III–IV than that of early stages I–II. Recently, many human miRNAs including but not limited to miR-26a, 29b, 141, 144, 205 and 221 were reported to target PTEN in various tumours^53^,^55^,^56^,^57^. However, we found that several of these miRNAs including miR-26a, 29b, 144 and 221 are significantly downregulated in NPC (see Supplementary Table 2), implying that EBV BART miRNAs in NPC may be more important than cellular miRNAs in the PTEN dosage regulation. Indeed, BART1 (both BART1-5p and BART1-3p) and BART7-3p target PTEN in NPC. It was noted that, based on bioinformatics analysis or PAR-CLIP predictions, several BART miRNAs (that is, BART9 and BART18-5p in NPC cells; BART2-5p, BART5, BART14* and BART21-3p in BC1 or AGS cells) would be possible to regulate PTEN^5^,^46^,^58^. However, their authenticity in epithelial carcinomas remains to be determined.

The article "Epstein–Barr virus-encoded microRNA BART1 induces tumour metastasis by regulating PTEN-dependent pathways in nasopharyngeal carcinoma" was retracted in 2025. Reasons: contaminated cell lines or tissues; duplicated images; overlap with earlier publications; unreliable data.

PTEN functions both as a dual specificity protein phosphatase and a lipid phosphatase^59^. The principal catalytic function of PTEN is to dephosphorylate phosphatidylinositol 3,4,5-trisphosphate (PIP3), a secondary messenger for Akt, to phosphatidylinositol 4,5-bisphosphate, thereby suppressing PI3K-Akt signalling by preventing PIP3-dependent processes such as the membrane recruitment and the activation of Akt and PKC. PTEN is also able to dephosphorylate protein substrates such as FAK and Shc, thus inhibiting the FAK-p130^Cas^ pathway^60^. Moreover, PTEN is capable of regulating MAPK–ERK1/2 signalling either by dephosphorylating Shc (resulting in the inactivation of Ras, Raf and ultimately ERK1/2) or by reducing PIP3-mediated activation of PKC and Akt (leading to the suppression of Raf, MEK and ERK1/2)^61^. In NPC, we found that BART1 significantly increased the phosphorylation levels of p-Akt, p-FAK, p130^Cas^, p-Shc and p-ERK1/2 in NPC cell lines. Importantly, such expression alterations also occurred *in vivo*, as revealed by IHC staining on tumour sections of xenografts and metastasized organs. Therefore, we concluded that EBV-miR-BART1 impels the migration and metastasis by targeting cellular PTEN and consequently activating PI3K-Akt, FAK-p130^Cas^ and MAPK–ERK1/2 pathways in NPC.

EMT, a fundamental biological process that enables polarized epithelial cells to convert mesenchymal-like cells, which includes the rearrangement of actin cytoskeleton and enhanced migratory and invasive capacity, is considered as the initial step of tumour metastasis^62^. FAK/p130^Cas^, PI3K/Akt and MAPK/ERK pathways were known to regulate EMT and promote cell migration^45^,^62^. In this study, we demonstrated that EBV-miR-BART1 in NPC cells significantly reduced the expression of E-cadherin, an important caretaker for the epithelial phenotype, but increased the expression of N-cadherin and vimentin, two goalkeepers for the mesenchymal phenotype. Consistently, downregulation of EBV-miR-BART1 increased the expression of E-cadherin but decreased the expression of N-cadherin and vimentin in NPC cell lines. IHC staining on tumour sections of xenografts and matastasized organs confirmed that BART1 decreased the expression of E-cadherin but increased the expression of vimentin *in vivo*. In clinical tumour samples, the expression of E-cadherin was reported downregulated and inversely correlated with lymph node metastasis of NPC^63^. Interestingly, we also found that BART1 modestly increased F-actin level and triggered actin cytoskeleton rearrangement in NPC cells apparently by activating FAK-p130^Cas^ and Shc-MEK-ERK1/2 pathways^59^,^60^,^61^. Collectively, our findings indicated that EBV-miR-BART1 increases cell motility and invasiveness by impelling EMT and increasing actin stress fibres in NPC cells.

The article "Epstein–Barr virus-encoded microRNA BART1 induces tumour metastasis by regulating PTEN-dependent pathways in nasopharyngeal carcinoma" was retracted in 2025. Reasons: contaminated cell lines or tissues; duplicated images; overlap with earlier publications; unreliable data.

In conclusion, we have demonstrated that EBV-miR-BART1 is highly expressed in NPC and closely associated with advanced stages of the patients. BART1 increased the cell migration and invasion of NPC *in vitro* and impelled the tumour metastasis *in vivo* by directly targeting PTEN. Reduction of PTEN dosage by BART1 activated PTEN-dependent pathways, compelled EMT and consequently increased the migration, invasion and metastasis of NPC (Fig. 7d). Reconstitution of PTEN expression rescued all phenotypes generated by BART1, highlighting the dominant role of PTEN in EBV-miR-BART-driven metastasis in NPC. Our findings provide new insights into the invasiveness and metastasis of NPC regulated by EBV and rational for the development of clinical intervention strategies for NPC.

## Methods

### Cell culture

Two EBV-negative NPC cell lines (CNE1 and 5-8F)^64^,^65^ and HEK293T cells were obtained from Cancer Research Institute Southern Medical University. Three EBV-positive NPC cell lines (HONE1-EBV, HK1-EBV and C666-1-EBV) were kindly provided by Professor S.-W. Tsao, University of Hong Kong. The NPC cell lines were cultured in RPMI-1640 (Invitrogen) supplemented with 10% newborn cow serum (NCS; Hyclone, Invitrogen), 100 U ml^−1^ penicillin and 100 μg ml^−1^ streptomycin, while HEK293T cells grew in Dulbecco's modified Eagle's medium (Invitrogen) with 10% NCS, 100 U ml^−1^ penicillin and 100 μg ml^−1^ streptomycin. All cells were maintained at 37 °C with 5% CO_2_.

### Patients and clinical tissue specimens

Primary NPC (no treatment before biopsy taking) and NP biopsies were collected from patients in Zhongshan People's Hospital, Guangdong, China. Informed written consent was obtained from all subjects and approval from the Ethics Committee of Zhongshan People's Hospital was obtained for research purposes in use of clinical materials. Twenty NPC and 20 NP specimens were used for microarray analysis and qRT–PCR validation (Supplementary Table 1) and another cohort containing 82 NPC specimens with TNM staging and 32 NP specimens were collected for the association analysis of EBV-miR-BART1 expression with pathological and clinical data (Supplementary Table 3). Only those NPC samples that contain >80% of homogeneous cancer cells on frozen cross-sections visualized by haematoxylin–eosin staining were included in this study. Staging was performed according to the China 1992 Fuzhou NPC staging system.

The article "Epstein–Barr virus-encoded microRNA BART1 induces tumour metastasis by regulating PTEN-dependent pathways in nasopharyngeal carcinoma" was retracted in 2025. Reasons: contaminated cell lines or tissues; duplicated images; overlap with earlier publications; unreliable data.

### qRT–PCR

Total RNA was extracted with TRIzol reagent (Invitrogen), complementary DNA (cDNA) was synthesized with the PrimeScript RT reagent Kit (TaKaRa, Dalian, China). qRT–PCR was performed in triplicate with SYBR Premix ExTaq (TaKaRa, Dalian, China). The primers used for amplification of the interested genes were listed in Supplementary Table 5. Quantification of EBV-miR-BART1 was conducted with TaqMan microRNA assays (Applied Biosystems). Mature miRNAs were reverse transcribed, and qRT–PCR was performed using All-in-One miRNA qRT–PCR Detection Kit following the manufacturer's protocol (GeneCopoeia). RPU6B and GAPDH were used for normalizing the expression of miRNA and mRNA, respectively. The fold changes were calculated by using the 2−ΔΔ*C*t method.

### MiRNA microarray analysis

MiRNA microarrays (CCDTM-miRNA850-V4p1.4) were kindly provided by Infectious Disease and Immunogenetics section, Department of Transfusion Medicine, Clinical Center, National Institutes of Health, USA. Total RNA was labelled by miRCURY LNA miRNA Power Labeling Kit (Exiqon Life Sciences, Vedbaek, Denmark) according to the manufacturer's instruction. The test sample and the reference were labelled with Hy5 and Hy3, respectively, and co-hybridized to the miRNA arrays. The hybridized arrays were scanned by LuxScanTM 10 K microarray Scanner (Capital Bio. Corporation, Beijing, China). The resulting data files were uploaded to the mAdb database. Any gene containing one of the follows was excluded: (1) <20% of expression data had at least a 1.5-fold-change in either direction from gene's median value; (2) per cent of data missing of filtered out exceeds 50%. Further analysis was done by using the BRB-Array Tools ( http://linus.nci.nih.gov/BRB-ArrayTools.html). Expression profile clustering and visualization were preformed with Cluster and Treeview software (Ernest Orlando Lawrence Berkeley National Laboratory, Berkeley, CA, USA). The raw data were deposited in GEO database (Superseries Accession Number: GSE42945).

### Lentivirus transductions

Lentiviral particles containing the GV209 expression vector encoding 282-nt pri-EBV-miR-BART1 precursor that produces both BART1-5p and BART1-3p (H1-miRNA-CMV-EGFP-BART1) and randomized flanking sequence control (H1-miRNA-CMV-EGFP-mock; Supplementary Fig. 8) were purchased from GeneChem (Shanghai, China) and transduced into NPC cells following the manufacturer's instructions. The virus-infected cells, being GFP positive, were sorted out by BD FACS Aria cell sorter after 72 h.

The article "Epstein–Barr virus-encoded microRNA BART1 induces tumour metastasis by regulating PTEN-dependent pathways in nasopharyngeal carcinoma" was retracted in 2025. Reasons: contaminated cell lines or tissues; duplicated images; overlap with earlier publications; unreliable data.

### Plasmid preparation and cell transfection

The expression vector GV230 ( http://www.genechem.com.cn) containing whole coding sequence of PTEN and the control vector GV170 were purchased from GeneChem (Shanghai, China). Plasmid DNAs were purified with TIANprep Mini Plasmid Kit (TIANGEN, China). Both CNE1-BART1 and 5-8F-BART1 cells were transfected with 200 ng plasmid DNA using Lipofectamine 2000 reagent (Invitrogen). Forty-eight hours post transfection, the cells were harvested for qRT–PCR and western blotting analyses. miRNA mimics or inhibitors (miRNA antisense oligonucleotides) were transfected at 50 nmol l^−1^ with Lipofectamine 2000 reagent (Invitrogen). The EBV-miR-BART1-5p mimic (5′-UCUUAGUGGAAGUGACGUGCUGUG-3′), EBV-miR-BART1-3p mimic (5′-UAGCACCGCUAUCCACUAUGUC-3′), EBV-miR-BART1-5p inhibitor (5′-CACAGCACGUCACUUCCACUAAGA-3′), EBV-miR-BART1-3p inhibitor (5′-GACAUAGUGGAUAGCGGUGCUA-3′) and associated nonspecific mimic (5′-UUGUACUACACAAAAGUACUG-3′) or inhibitor (5′-CAGUACUUUUGUGUAGUACAA-3′) controls were synthesized by GenePharma, Shanghai, China.

### Transwell migration and Boyden chamber invasion assays

For the transwell migration assay, 10^5^ cells in 100 μl of serum-free DMEM media were triplicate seeded in each fibronectin-coated polycarbonate membrane insert in a transwell apparatus (Corning). 600 μl of 10% NCS in DMEM was added to the bottom chamber. CNE1 and 5-8F cells were incubated at 37 °C for 18 h and 12 h, respectively. The inserts were washed twice with prewarmed PBS. Cells adhered on the lower surface were fixed with 100% methanol at RT for 15 min and stained with hematoxylin for 15 min. Cell numbers in six predetermined fields in each replicate were counted under the microscope (NiKon ECLPSE 80i system; × 200). All assays were independently repeated at least for three times. Cell invasion assays were performed as the migration assay except the transwell membrane was precoated with 24 mg ml^−1^ Matrigel (R&D Systems) and the cells were incubated for 24 and 18 h, respectively.

### Western blotting

Western blotting analyses were performed by using standard methods. In brief, cells were harvested and lysed in the RIPA buffer containing protease inhibitors (Sigma-Aldrich) and phosphatase inhibitors (Keygen, China). Proteins were separated by SDS–polyacrylamide gel electrophoresis gels, and blotted onto PVDF membrane (Millipore). The membrane was probed with the first antibody listed in Supplementary Table 6 and then with the peroxidase-conjugated secondary antibody. GAPDH was used as a protein loading control. Western blotting bands were visualized by eECL Western Blot Kit (CWBIO Technology) and captured with ChemiDocTM CRS+ Molecular Imager (Bio-Rad). All blots in figures were accompanied by the locations of molecular weight/size markers. Original blotting images for the key components of PTEN-dependent pathways and EMT were shown in Supplementary Fig. 9.

The article "Epstein–Barr virus-encoded microRNA BART1 induces tumour metastasis by regulating PTEN-dependent pathways in nasopharyngeal carcinoma" was retracted in 2025. Reasons: contaminated cell lines or tissues; duplicated images; overlap with earlier publications; unreliable data.

### Tumour xenografts in nude mice

Animal experiments were approved by the Ethical Committee for Animal Research of Southern Medical University (protocol number: 2011-020) and conducted based on the state guidelines from the Ministry of Science and Technology of China. All nude mice (4–5 weeks old, female) were purchased from the Central Animal Facility of Southern Medical University. To assess tumour growth, 200 μl of 5-8F-BART1 cells or mock control cells (10^7^) was subcutaneously injected into the left or right side on the back of each mouse (seven mice per group). The tumour sizes were measured regularly and calculated using the formula=0.52 × L × W^2^ where L and W are the long and short diameter of the tumour, respectively.

We chose the well-established mouse model to evaluate tumour metastasis^43^,^44^. Under the anaesthesia by peritoneal injection of 1% pentobarbital sodium, a small cut on the abdominal region was made. The mouse liver was gently pushed out of abdominal cavity and 50 μl of 5-8F cells (2 × 10^6^) was then injected underneath the liver envelope. The liver was then pushed back into abdominal cavity after lightly pressed the pinhole with alcohol cotton balls for two minutes. All mice (seven per group) were killed on day 21 after transplantation, or earlier if the mouse reached the ethical endpoint. Whole bodies, freshly dissected tumours and internal organs including lungs, livers and lymph nodes were collected for fluorescence imaging with the LT-9MACIMSYSPLUS whole-body imaging system (Encinitas, CA)^29^. Tumour tissues were fixed in 4% paraformaldehyde for 48 h and transferred to gradient ethanol. Tumours were embedded in paraffin, sectioned with LeiCa RM2235 and processed for histological examinations.

### F-actin staining and confocal microscope examinations

F-actin staining was monitored by Rhodamine-phalloidin (5 μg ml^−1^) and 4′,6-diamidino-2-phenylindole (DAPI) (0.1 μg ml^−1^) staining according to the manufacturer's instructions. In brief, the cells were seeded on sterile coverslips with monolayer on the day before staining. Cells were then washed with prewarmed PBS twice, fixed with 4% paraformaldehyde in PBS for 10 min and washed with PBS three times, each for 5 min. Cells were then permeablized with cold 100% acetone for 5 min, washed and treated with 1% bovine serum albumin/PBS/0.1% azide for 30 min for blocking nonspecific binding. Subsequently, cells were stained with Rhodamine-phalloidin at RT for 30 min, washed with PBS twice, stained for nuclei with DAPI for 1 min. The coverslips were mounted on slides using anti-fade mounting medium. Confocal images were acquired on the OLYMPUS confocal micrograph system, and analysed with FV10-ASW1.7 viewer software (Olympus).

The article "Epstein–Barr virus-encoded microRNA BART1 induces tumour metastasis by regulating PTEN-dependent pathways in nasopharyngeal carcinoma" was retracted in 2025. Reasons: contaminated cell lines or tissues; duplicated images; overlap with earlier publications; unreliable data.

### IF assays

Cells were cultured on coverslips overnight, fixed with 4% formaldehyde in PBS for 15 min at 4 °C and then permeabilized with 0.5% Triton-X-100 in PBS for 30 min. Subsequently, cells were blocked for nonspecific binding with 5% milk in TBS and Tween-20 (TBST) at RT for 30 min, incubated with PTEN-specific antibody (1:100, Bioworld) at 4 °C overnight. The cells were incubated with Alexa Fluor 488 goat anti-rabbit IgG (1:500, Sigma-Aldrich) at 37 °C for 1 h. The coverslips were mounted on slides using anti-fade mounting medium with DAPI. IF images were acquired on Nikon ECLIPSE 80i microscope (Nikon).

### IHC staining

Paraffin sections prepared from *in vivo* experiments were applied to IHC staining for the detection of protein levels of PTEN and some key components of PTEN-pathways. The indirect streptavidin-peroxidase method was used^29^. All antibodies used for IHC were listed in Supplementary Table 6. The stained results were reviewed and scored by two pathologists independently 66. In brief, the intensity of immunostaining was scored as negative (0), weak (1), medium (2) and strong (3). The extent of staining, defined as the per cent of positive staining cells, was scored as 1 (≤10%), 2 (11–50%), 3 (51–75%) and 4 (>75%). An overall expression score, ranging from 0 to 12, was obtained by multiplying the score of intensity and that of extent. The final staining score was presented as negative (overall score of (0), 1+ (overall score of 1–3), 2+ (overall score of 4) or 3+ (overall score of ≥5).

### RNA-deep sequencing

RNA-deep sequencing was performed and analysed in BGI-Shenzhen of China. In brief, mRNAs were isolated from the DNase-treated total RNAs with the Dynabeads mRNA Purification Kit (Life Technologies). According to the manufacturer's instructions, the mRNAs were fragmented with divalent cations and converted to single-strand cDNA with random hexamer primers and Superscript II reverse transcriptase (Life Technologies). The second strand of cDNA was generated by RNase H (Enzymatics) and DNA polymerase. cDNA products were purified by Ampure beads XP (Beckman). After converting the overhangs into blunt ends using T4 DNA polymerase and Klenow DNA polymerase, extra ‘A' base was added to the 3′-end of cDNA by Klenow enzyme. Sequencing adapters were then ligated to the end of cDNA by T4 DNA Ligase (Enzymatics). The fragments of 200 bp were selected by Ampure beads XP (Beckman) and enriched by 12 cycles of PCR. The PCR products were loaded into flowcell to generate clusters and then sequenced by Hiseq 2000 (Illumina). The resulting data were deposited in GEO database (Accession Number: GSE42945). Selected results were shown in Supplementary Table 4.

The article "Epstein–Barr virus-encoded microRNA BART1 induces tumour metastasis by regulating PTEN-dependent pathways in nasopharyngeal carcinoma" was retracted in 2025. Reasons: contaminated cell lines or tissues; duplicated images; overlap with earlier publications; unreliable data.

### MiRNA target predictions

EBV-miR-BART1 candidate targets were initially obtained from the RNA-deep sequencing in BGI-Shenzhen of China (Supplementary Table 4) and then enriched with literature retrieval. The RNAhybrid programme ( http://bibiserv.techfak.uni-bielefeld.de/rnahybrid/submission.html) was used to predict duplex complementation between human PTEN 3′-UTR and EBV-miR-BART1-5p or EBV-miR-BART1-3p.

### Luciferase reporter assays

The MiTarget microRNA 3′-UTR target vector (pEZX-MT01) containing full-length 3′-UTR of PTEN with two binding sites for EBV-miR-BART1-5p and EBV-miR-BART1-3p (wild-type 3′-UTR) was produced by GeneCopoeia. Two mutant sites (mut1 and mut2) in PTEN 3′-UTR were then generated by site-directed mutagenesis with KOD-Plus-Mutagenesis Kit (SMK-101, Toyobo C. Ltd). For luciferase reporter assays, wt or mut 3′-UTR vector was co-transfected with EBV-miR-BART1 mimic or nonspecific mimic control (Genepharma) into HEK 293 T cells, respectively. Luciferase activity was measured 48 h after transfection using Luc-Pair miR Luciferase Assay Kit (GeneCopoeia) on Panomics Luminometer.

### Statistical analysis

All experiments were performed in triplicate. Data shown are mean±s.e.m. (unless otherwise specified) from at least three independent experiments. SPSS 16.0 software was used for statistical analyses. Differences were considered to be statistically significant at values of *P*<0.05 by Student's *t*-test for two groups, one-way ANOVA (analysis of variance) analysis for multiple groups and parametric generalized linear model with random effects for tumour growth. Correlation was analysed with two-tailed Spearman's correlation analysis. Single, double and triple asterisks indicate statistical significance—*P<0.05, **P<0.01 and ***P<0.001.

## Additional information

The micrRNA microarray data were deposited in the GEO database under Superseries Accession Number: GSE42945. The RNA sequencing data have been in deposited in the GEO database under accession code GSE42945).

**How to cite this article:** Cai, L. *et al.* Epstein–Barr virus-encoded microRNA BART1 induces tumour metastasis by regulating PTEN-dependent pathways in nasopharyngeal carcinoma. *Nat. Commun.* 6:7353 doi: 10.1038/ncomms8353 (2015).

## Supplementary Material

Supplementary Information Supplementary Figures 1-9 and Supplementary Tables 1-6

## Figures and Tables

**Figure 1:** EBV-miR-BART1 is highly expressed in NPC and associated with clinicopathological features. (**a**) MiRNA expression profile microarray screening. Supervised hierarchical cluster analysis of 69 miRNAs that were differentially expressed between 20 NPC and 20 NP biopsies (universal test *P*<0.005, fold-change >1.5, false discovery rate <0.05). Left: heatmap of the 69 miRNAs differentially expressed between NPC and NP samples. Red represents upregulated miRNAs and blue for downregulated miRNAs. Right-up: the top seven upregulated EBV BART miRNAs clustered together. Right-down: a volcano plot for the visualization of differentially expressed miRNAs with significance cut off *P*<0.005 and fold-change ≥1.5 symmetrically in NPC compared with NP. The top 11 upregulated EBV BART miRNAs in NPC were highlighted by a red dot-line square. (**b**) EBV-miR-BART1 was highly expressed in late pathological stages of NPC. The expression of EBV-miR-BART1 in a separated cohort of 82 NPC samples was determined by qRT–PCR. RPU6B was used for normalizing the expression of BART1-5p or BART1-3p. Student's *t*-test, mean±s.e.m., *P<0.05, **P<0.01. (**c**) EBV-miR-BART1 was highly expressed in advanced clinical stages of NPC. Both BART1-5p and BART1-3p were highly expressed in advanced clinical stages (III–IV) compared with that of early clinical stages (I–II). Student's *t*-test, mean±s.e.m., *P<0.05, **P<0.01.

The article "Epstein–Barr virus-encoded microRNA BART1 induces tumour metastasis by regulating PTEN-dependent pathways in nasopharyngeal carcinoma" was retracted in 2025. Reasons: contaminated cell lines or tissues; duplicated images; overlap with earlier publications; unreliable data.

**Figure 2:** EBV-miR-BART1 propels cell migration and invasion *in vitro* and tumour metastasis of NPC *in vivo*. (**a**) Transwell migration assays. Upregulation of BART1 miRNA increased the cell migration of both CNE1-BART1 and 5-8F-BART1 compared with relative mock cells. Student's *t*-test. (**b**) Boyden chamber invasion assays. Upregulation of BART1 miRNA increased the cell invasion of both CNE1-BART1 and 5-8F-BART1 compared with relative mock cells. Student's *t*-test. (**c**) Downregulation of BART1 miRNA by the BART1 inhibitor decreased the cell migration of both CNE1-BART1 and 5-8F-BART1. One-way ANOVA and Dunnett's multiple comparison test. (**d**) Downregulation of BART1 miRNA by the BART1 inhibitor decreased the cell invasion of both CNE1-BART1 and 5-8F-BART1. One-way ANOVA and Dunnett's multiple comparison test. (**e**) Xenograft tumours collected on day 21 post subcutaneous implantation of 5-8F cells. Upregulation of BART1 increased the tumour growth in nude mice (5-8F-BART1 versus 5-8F-mock). (**f**) Tumour growth curves. Upregulation of BART1 increased the tumour growth in nude mice (5-8F-BART1 versus 5-8F-mock). *N*=7, parametric generalized linear model with random effects. (**g**) Representative GFP images of tumour metastasis. Upregulation of BART1 increased the tumour metastasis in lung, liver and lymph nodes. *N*=7. (**h**) Upregulation of BART1 increased the tumour metastasis in lung, liver and lymph nodes. *N*=7, *χ*^2^-test for left panel and Student's *t*-test for right panel. Original magnification, × 200; scale bar, 25 μm. Mean±s.e.m., *N*=3, *P<0.05, **P<0.01, ***P<0.001.

The article "Epstein–Barr virus-encoded microRNA BART1 induces tumour metastasis by regulating PTEN-dependent pathways in nasopharyngeal carcinoma" was retracted in 2025. Reasons: contaminated cell lines or tissues; duplicated images; overlap with earlier publications; unreliable data.

**Figure 3:** EBV-miR-BART1 targets tumour suppressor PTEN in NPC. (**a**) Development of the integrated strategy for discovering targeted genes of EBV-miR-BART1. (**b**) Bioinformatics predictions of two binding sites by BART1-5p and BART1-3p in PTEN 3′-UTR region. Wild-type (wt) and two mutant sequences are indicated. (**c**) Luciferase reporter assays. HEK293T cells were co-transfected with wt or mutated PTEN 3′-UTR and the BART1 mimic (either b1-5p for BART1-5p or b1-3p for BART1-3p) or nonspecific mimic control (NC). Relative repression of firefly luciferase expression was standardized to a transfection control. One-way ANOVA and Dunnett's multiple comparison test. (**d**) The expression of PTEN in two cell lines and tumour sections of 5-8F xenografts and metastasized organs. Up panels are representatives of IF staining for PTEN (red) in both CNE1-BART1 and 5-8F-BART1 cells and relative mock control cells. Nuclei were stained with DAPI (blue). Low panels are the representatives of IHC staining for PTEN in metastasized tumours (liver and lymph node) from 5-8F tumours. Original magnification, × 400; scale bar, top panel 10 μm, bottom panel 25 μm. (**e**) The expression of PTEN at mRNA level in 32 NP and 82 NPC specimens determined by qRT–PCR. Left panel: significant downregulation of PTEN in N2–3 pathological stages compared with that of N0–1 stages or with NP. Right panel: significant downregulation of PTEN in advanced clinical stages (III–IV) compared with early clinical stages (I–II) or compared with NP. (**f**) Reverse correlation of the expression EBV-miR-BART1 and PTEN. Left: BART1-5p versus PTEN, right: BART1-3p versus PTEN. Two-tailed Spearman's correlation analysis. One-way ANOVA and Dunnett's multiple comparison test. Mean±s.e.m., **P<0.01, ***P<0.001.

**Figure 4:** EBV-miR-BART1 activates PTEN-dependent pathways. (**a**) Upregulation of EBV-miR-BART1 decreased the protein expression of PTEN but increased the expression of p-Akt, FAK, p-FAK, p130^Cas^, p-Shc and p-ERK1/2 in both CNE1-BART1 and 5-8F-BART1 cells. GAPDH was a protein loading control. (**b**) Downregulation of EBV-miR-BART1 by the BART1 miRNA inhibitor increased the protein expression of PTEN but decreased the protein phosphorylation of p-Akt, p-FAK, p130^Cas^, p-Shc and p-ERK1/2 in both CNE1-BART1 and 5-8F-BART1 cells. (**c**) Upregulation of EBV-miR-BART1 increased the phosphorylation levels of p-Akt, p130^Cas^, p-Shc and p-ERK1/2 in tumour sections of 5-8F metastasized organs revealed by IHC staining (5-8F-BART1 versus 5-8F-mock). Original magnification, × 400; scale bar, 25 μm. One-way ANOVA and Dunnett's multiple comparison test. Mean±s.e.m., *N*=5, **P<0.01.

The article "Epstein–Barr virus-encoded microRNA BART1 induces tumour metastasis by regulating PTEN-dependent pathways in nasopharyngeal carcinoma" was retracted in 2025. Reasons: contaminated cell lines or tissues; duplicated images; overlap with earlier publications; unreliable data.

**Figure 5:** EBV-miR-BART1 compels EMT. (**a**) Upregulation of EBV-miR-BART1 expression by retrivirus transductions decreased the protein level of E-cadherin but increased the expression level of N-cadherin and vimentin in both CNE1-BART1 and 5-8F-BART1 cells. (**b**) Downregulation of EBV-miR-BART1 expression by the BART1 miRNA inhibitor increased the protein level of E-cadherin but decreased the expression level of N-cadherin and vimentin in both CNE1-BART1 and 5-8F-BART1 cells. (**c**) Upregulation of EBV-miR-BART1 decreased the expression of E-cadherin but increased the expression of vimentin in tumour sections of 5-8F metastasized organs revealed by IHC staining (5-8F-BART1 versus 5-8F-mock). Original magnification, × 400; scale bar, 25 μm. One-way ANOVA and Dunnett's multiple comparison test. Mean±s.e.m., *N*=5, *P<0.05, **P<0.01. (**d**) EBV-miR-BART1 enhanced the rearrangement of actin cytoskeleton. Stress fibres and actin filaments were visualized by Rhodamine-phalloidin staining (red) in NPC cells tranduced with lentivirus (green for GFP). Nuclei were stained with DAPI (blue). Upregulation of BART1 modestly increased F-actin expression (red) and actin stress fibres throughout the BART1-expressing cells compared with the control cells in which the actin bundles were predominantly localized underneath cell membranes. Original magnification, × 1,200; scale bar, 5 μm.

**Figure 6:** Reconstitution of PTEN rescues the phenotypes generated by EBV-miR-BART1. (**a**) Reconstitution of PTEN reduced the cell migration of both CNE1-BART1 and 5-8F-BART1 cells. (**b**) Reinstallation of PTEN reduced the cell invasion of both CNE1-BART1 and 5-8F-BART1 cells. (**c**) Restitution of PTEN decreased the phosphorylation levels of p-Akt, p-FAK, p130^Cas^, p-Shc and p-ERK1/2 in both CNE1-BART1 and 5-8F-BART1 cells (PTEN versus NC). (**d**) Restoration of PTEN dosage increased the expression of E-cadherin but decreased the expression of either N-cadherin or vimentin in both CNE1-BART1 and 5-8F-BART1 cells (PTEN versus NC). Original magnification, × 200; scale bar, 25 μm. Student's *t*-test, mean±s.e.m., *N*=3. ***P<0.001.

**Figure 7:** Downregulation of EBV-miR-BART1 attenuates cell mobility, PTEN-dependent signalling and EMT of EBV-positive NPC cells. (**a**) Downregulation of EBV-miR-BART1 by the BART1 inhibitor decreased the cell migration of HONE1-EBV-positive cells. (**b**) Downregulation of EBV-miR-BART1 by the BART1 inhibitor reduced the cell invasion of HONE1-EBV-positive cells. (**c**) Downregulation of EBV-miR-BART1 by the BART1 inhibitor increased the protein expressions of PTEN and E-cadherin but decreased the expressions of p-Akt, p-FAK, p-ERK1/2, N-cadherin and vimentin in HONE1-EBV-positive cells. (**d**) A proposed model demonstrating the role of EBV-miR-BART1 in NPC metastasis. EBV latently infected >90% of human population. Under certain circumstances, particularly at advanced stages of NPC, EBV produced a great amount of BART miRNAs including EVB-miR-BART1. BART1 miRNA directly targets host PTEN, one of the major tumour suppressor and reduces the PTEN dosage, resulting in the activation of PTEN-dependent pathways including PI3K-Akt, FAK-p130^Cas^ and Shc-MAPK/ERK1/2 signalling. Consequently, BART1 miRNA compels actin cytoskeleton rearrangement and EMT, thus impelling the migration, invasion and metastasis of NPC. Original magnification, × 200; scale bar, 25 μm. One-way ANOVA and Dunnett's multiple comparison test, mean±s.e.m., *N*=3, ***P<0.001.

The article "Epstein–Barr virus-encoded microRNA BART1 induces tumour metastasis by regulating PTEN-dependent pathways in nasopharyngeal carcinoma" was retracted in 2025. Reasons: contaminated cell lines or tissues; duplicated images; overlap with earlier publications; unreliable data.

## References

[b1] WeiW. I. & ShamJ. S. Nasopharyngeal carcinoma. Lancet 365, 2041–2054 (2005).1595071810.1016/S0140-6736(05)66698-6

[b2] LoK. W., ChungG. T. & ToK. F. Deciphering the molecular genetic basis of NPC through molecular, cytogenetic, and epigenetic approaches. Semin. Cancer Biol. 22, 79–86 (2012).2224547310.1016/j.semcancer.2011.12.011

[b3] KutokJ. L. & WangF. Spectrum of Epstein-Barr virus-associated diseases. Annu. Rev. Pathol. 1, 375–404 (2006).1803912010.1146/annurev.pathol.1.110304.100209

[b4] TsaoS. W., TsangC. M., ToK. F. & LoK. W. The role of Epstein-Barr virus in epithelial malignancies. J. Pathol. 235, 323–333 (2015).2525173010.1002/path.4448PMC4280676

[b5] MarquitzA. R., MathurA., ShairK. H. & Raab-TraubN. Infection of Epstein-Barr virus in a gastric carcinoma cell line induces anchorage independence and global changes in gene expression. Proc. Natl Acad. Sci. USA 109, 9593–9598 (2012).2264760410.1073/pnas.1202910109PMC3386136

[b6] Raab-TraubN. Novel mechanisms of EBV-induced oncogenesis. Curr. Opin. Virol. 2, 453–458 (2012).2285811810.1016/j.coviro.2012.07.001PMC4617531

[b7] BartelD. P. MicroRNAs: genomics, biogenesis, mechanism, and function. Cell 116, 281–297 (2004).1474443810.1016/s0092-8674(04)00045-5

[b8] Esquela-KerscherA. & SlackF. J. Oncomirs - microRNAs with a role in cancer. Nat. Rev. Cancer 6, 259–269 (2006).1655727910.1038/nrc1840

[b9] PfefferS. *et al.* Identification of virus-encoded microRNAs. Science 304, 734–736 (2004).1511816210.1126/science.1096781

The article "Epstein–Barr virus-encoded microRNA BART1 induces tumour metastasis by regulating PTEN-dependent pathways in nasopharyngeal carcinoma" was retracted in 2025. Reasons: contaminated cell lines or tissues; duplicated images; overlap with earlier publications; unreliable data.

[b10] ChenS. J. *et al.* Characterization of Epstein-Barr virus miRNAome in nasopharyngeal carcinoma by deep sequencing. PLoS ONE 5, e12745 (2010).2086221410.1371/journal.pone.0012745PMC2942828

[b11] KuzembayevaM., HayesM. & SugdenB. Multiple functions are mediated by the miRNAs of Epstein-Barr virus. Curr. Opin. Virol. 7C, 61–65 (2014).2481466610.1016/j.coviro.2014.04.003PMC4149930

[b12] LoA. K., DawsonC. W., JinD. Y. & LoK. W. The pathological roles of BART miRNAs in nasopharyngeal carcinoma. J. Pathol. 227, 392–403 (2012).2243106210.1002/path.4025

[b13] PrattZ. L., KuzembayevaM., SenguptaS. & SugdenB. The microRNAs of Epstein-Barr Virus are expressed at dramatically differing levels among cell lines. Virology 386, 387–397 (2009).1921713510.1016/j.virol.2009.01.006PMC2763627

[b14] ZengZ. *et al.* Regulation network and expression profiles of Epstein-Barr virus-encoded microRNAs and their potential target host genes in nasopharyngeal carcinomas. Sci. China Life Sci. 57, 315–326 (2014).2453245710.1007/s11427-013-4577-y

[b15] QiuJ. *et al.* A novel persistence associated EBV miRNA expression profile is disrupted in neoplasia. PLoS Pathog. 7, e1002193 (2011).2190109410.1371/journal.ppat.1002193PMC3161978

[b16] MarquitzA. R., MathurA., ChughP. E., DittmerD. P. & Raab-TraubN. Expression profile of microRNAs in Epstein-Barr virus-infected AGS gastric carcinoma cells. J. Virol. 88, 1389–1393 (2014).2422784910.1128/JVI.02662-13PMC3911632

[b17] ImigJ. *et al.* microRNA profiling in Epstein-Barr virus-associated B-cell lymphoma. Nucleic Acids Res. 39, 1880–1893 (2011).2106281210.1093/nar/gkq1043PMC3061055

[b18] CosmopoulosK. *et al.* Comprehensive profiling of Epstein-Barr virus microRNAs in nasopharyngeal carcinoma. J. Virol. 83, 2357–2367 (2009).1909185810.1128/JVI.02104-08PMC2643705

[b19] AmorosoR. *et al.* Quantitative studies of Epstein-Barr virus-encoded microRNAs provide novel insights into their regulation. J. Virol. 85, 996–1010 (2011).2106824810.1128/JVI.01528-10PMC3020024

[b20] YangH. J. *et al.* Comprehensive profiling of Epstein-Barr virus-encoded miRNA species associated with specific latency types in tumor cells. Virol. J. 10, 314 (2013).2416101210.1186/1743-422X-10-314PMC4231337

[b21] CaiX. *et al.* Epstein-Barr virus microRNAs are evolutionarily conserved and differentially expressed. PLoS Pathog. 2, e23 (2006).1655729110.1371/journal.ppat.0020023PMC1409806

[b22] Kim doN. *et al.* Expression of viral microRNAs in Epstein-Barr virus-associated gastric carcinoma. J. Virol. 81, 1033–1036 (2007).1707930010.1128/JVI.02271-06PMC1797424

[b23] LoA. K. *et al.* Modulation of LMP1 protein expression by EBV-encoded microRNAs. Proc. Natl Acad. Sci. USA 104, 16164–16169 (2007).1791126610.1073/pnas.0702896104PMC2042179

The article "Epstein–Barr virus-encoded microRNA BART1 induces tumour metastasis by regulating PTEN-dependent pathways in nasopharyngeal carcinoma" was retracted in 2025. Reasons: contaminated cell lines or tissues; duplicated images; overlap with earlier publications; unreliable data.

[b24] ZhuJ. Y. *et al.* Identification of novel Epstein-Barr virus microRNA genes from nasopharyngeal carcinomas. J. Virol. 83, 3333–3341 (2009).1914471010.1128/JVI.01689-08PMC2655542

[b25] ChoyE. Y. *et al.* An Epstein-Barr virus-encoded microRNA targets PUMA to promote host cell survival. J. Exp. Med. 205, 2551–2560 (2008).1883854310.1084/jem.20072581PMC2571930

[b26] BarthS. *et al.* Epstein-Barr virus-encoded microRNA miR-BART2 down-regulates the viral DNA polymerase BALF5. Nucleic Acids Res. 36, 666–675 (2008).1807319710.1093/nar/gkm1080PMC2241876

[b27] LungR. W. *et al.* Modulation of LMP2A expression by a newly identified Epstein-Barr virus-encoded microRNA miR-BART22. Neoplasia 11, 1174–1184 (2009).1988195310.1593/neo.09888PMC2767219

[b28] NachmaniD., Stern-GinossarN., SaridR. & MandelboimO. Diverse herpesvirus microRNAs target the stress-induced immune ligand MICB to escape recognition by natural killer cells. Cell Host Microbe 5, 376–385 (2009).1938011610.1016/j.chom.2009.03.003

[b29] LyuX. *et al.* TGFbetaR2 is a major target of miR-93 in nasopharyngeal carcinoma aggressiveness. Mol. Cancer 13, 51 (2014).2460663310.1186/1476-4598-13-51PMC4016586

[b30] YeY. *et al.* EBV-miR-BART1 is involved in regulating metabolism-associated genes in nasopharyngeal carcinoma. Biochem. Biophys. Res. Commun. 436, 19–24 (2013).2368514710.1016/j.bbrc.2013.05.008

[b31] BoyerinasB., ParkS. M., HauA., MurmannA. E. & PeterM. E. The role of let-7 in cell differentiation and cancer. Endocr. Relat. Cancer 17, F19–F36 (2010).1977903510.1677/ERC-09-0184

[b32] ChenH. C. *et al.* MicroRNA deregulation and pathway alterations in nasopharyngeal carcinoma. Br. J. Cancer 100, 1002–1011 (2009).1929381210.1038/sj.bjc.6604948PMC2661776

[b33] OuzounovaM. *et al.* MicroRNA miR-30 family regulates non-attachment growth of breast cancer cells. BMC Genomics 14, 139 (2013).2344540710.1186/1471-2164-14-139PMC3602027

[b34] LuJ. *et al.* MiR-26a inhibits cell growth and tumorigenesis of nasopharyngeal carcinoma through repression of EZH2. Cancer Res. 71, 225–233 (2011).2119980410.1158/0008-5472.CAN-10-1850

[b35] BorralhoP. M. *et al.* miR-143 overexpression impairs growth of human colon carcinoma xenografts in mice with induction of apoptosis and inhibition of proliferation. PLoS ONE 6, e23787 (2011).2190113510.1371/journal.pone.0023787PMC3162002

[b36] ReidG. *et al.* Restoring expression of miR-16: a novel approach to therapy for malignant pleural mesothelioma. Ann. Oncol. 24, 3128–3135 (2013).2414881710.1093/annonc/mdt412

[b37] CheungC. C. *et al.* miR-31 is consistently inactivated in EBV-associated nasopharyngeal carcinoma and contributes to its tumorigenesis. Mol. Cancer 13, 184 (2014).2509867910.1186/1476-4598-13-184PMC4127521

The article "Epstein–Barr virus-encoded microRNA BART1 induces tumour metastasis by regulating PTEN-dependent pathways in nasopharyngeal carcinoma" was retracted in 2025. Reasons: contaminated cell lines or tissues; duplicated images; overlap with earlier publications; unreliable data.

[b38] ShenQ. *et al.* MiR-101 functions as a tumor suppressor by directly targeting nemo-like kinase in liver cancer. Cancer Lett. 344, 204–211 (2014).2418945810.1016/j.canlet.2013.10.030

[b39] MeiJ., BachooR. & ZhangC. L. MicroRNA-146a inhibits glioma development by targeting Notch1. Mol. Cell. Biol. 31, 3584–3592 (2011).2173028610.1128/MCB.05821-11PMC3165557

[b40] ItoM. *et al.* MicroRNA-150 inhibits tumor invasion and metastasis by targeting the chemokine receptor CCR6, in advanced cutaneous T-cell lymphoma. Blood 123, 1499–1511 (2014).2438554010.1182/blood-2013-09-527739

[b41] TsurutaT. *et al.* miR-152 is a tumor suppressor microRNA that is silenced by DNA hypermethylation in endometrial cancer. Cancer Res. 71, 6450–6462 (2011).2186875410.1158/0008-5472.CAN-11-0364

[b42] XuT. *et al.* MicroRNA-195 suppresses tumorigenicity and regulates G1/S transition of human hepatocellular carcinoma cells. Hepatology 50, 113–121 (2009).1944101710.1002/hep.22919

[b43] LiuT. *et al.* An imageable metastatic treatment model of nasopharyngeal carcinoma. Clin. Cancer Res. 13, 3960–3967 (2007).1760673010.1158/1078-0432.CCR-07-0089

[b44] YangM. *et al.* Direct external imaging of nascent cancer, tumor progression, angiogenesis, and metastasis on internal organs in the fluorescent orthotopic model. Proc. Natl Acad. Sci. USA 99, 3824–3829 (2002).1189129410.1073/pnas.052029099PMC122608

[b45] LamouilleS., XuJ. & DerynckR. Molecular mechanisms of epithelial-mesenchymal transition. Nat. Rev. Mol. Cell Biol. 15, 178–196 (2014).2455684010.1038/nrm3758PMC4240281

[b46] WongA. M., KongK. L., TsangJ. W., KwongD. L. & GuanX. Y. Profiling of Epstein-Barr virus-encoded microRNAs in nasopharyngeal carcinoma reveals potential biomarkers and oncomirs. Cancer 118, 698–710 (2012).2172099610.1002/cncr.26309

[b47] LeiT. *et al.* Targeting of DICE1 tumor suppressor by Epstein-Barr virus-encoded miR-BART3* microRNA in nasopharyngeal carcinoma. Int. J. Cancer 133, 79–87 (2013).2328082310.1002/ijc.28007

[b48] RileyK. J. *et al.* EBV and human microRNAs co-target oncogenic and apoptotic viral and human genes during latency. EMBO J. 31, 2207–2221 (2012).2247320810.1038/emboj.2012.63PMC3343464

[b49] HsuC. Y. *et al.* The Epstein-Barr virus-encoded microRNA MiR-BART9 promotes tumor metastasis by targeting E-cadherin in nasopharyngeal carcinoma. PLoS Pathog. 10, e1003974 (2014).2458617310.1371/journal.ppat.1003974PMC3937311

[b50] CaiL. M. *et al.* EBV-miR-BART7-3p promotes the EMT and metastasis of nasopharyngeal carcinoma cells by suppressing the tumor suppressor PTEN. Oncogene (2014).10.1038/onc.2014.34125347742

The article "Epstein–Barr virus-encoded microRNA BART1 induces tumour metastasis by regulating PTEN-dependent pathways in nasopharyngeal carcinoma" was retracted in 2025. Reasons: contaminated cell lines or tissues; duplicated images; overlap with earlier publications; unreliable data.

[b51] SalmenaL., CarracedoA. & PandolfiP. P. Tenets of PTEN tumor suppression. Cell 133, 403–414 (2008).1845598210.1016/j.cell.2008.04.013

[b52] SongL. B. *et al.* The polycomb group protein Bmi-1 represses the tumor suppressor PTEN and induces epithelial-mesenchymal transition in human nasopharyngeal epithelial cells. J. Clin. Invest. 119, 3626–3636 (2009).1988465910.1172/JCI39374PMC2786794

[b53] ZhangL. Y. *et al.* MicroRNA-144 promotes cell proliferation, migration and invasion in nasopharyngeal carcinoma through repression of PTEN. Carcinogenesis 34, 454–463 (2013).2312522010.1093/carcin/bgs346

[b54] ChenQ., SamaranayakeL. P., ZhouH. & XiaoL. Homozygous deletion of the PTEN tumor-suppressor gene is not a feature in oral squamous cell carcinoma. Oral. Oncol. 36, 95–99 (2000).1088992710.1016/s1368-8375(99)00068-8

[b55] QuC. *et al.* MiR-205 determines the radioresistance of human nasopharyngeal carcinoma by directly targeting PTEN. Cell Cycle 11, 785–796 (2012).2237467610.4161/cc.11.4.19228PMC3356830

[b56] SongM. S., SalmenaL. & PandolfiP. P. The functions and regulation of the PTEN tumour suppressor. Nat. Rev. Mol. Cell Biol. 13, 283–296 (2012).2247346810.1038/nrm3330

[b57] ZhangL. *et al.* microRNA-141 is involved in a nasopharyngeal carcinoma-related genes network. Carcinogenesis 31, 559–566 (2010).2005392710.1093/carcin/bgp335

[b58] GottweinE. *et al.* Viral microRNA targetome of KSHV-infected primary effusion lymphoma cell lines. Cell Host Microbe 10, 515–526 (2011).2210016510.1016/j.chom.2011.09.012PMC3222872

[b59] YamadaK. M. & ArakiM. Tumor suppressor PTEN: modulator of cell signaling, growth, migration and apoptosis. J. Cell Sci. 114, 2375–2382 (2001).1155974610.1242/jcs.114.13.2375

[b60] GuJ. *et al.* Shc and FAK differentially regulate cell motility and directionality modulated by PTEN. J. Cell Biol. 146, 389–403 (1999).1042709210.1083/jcb.146.2.389PMC2156182

[b61] ChetramM. A. & HintonC. V. PTEN regulation of ERK1/2 signaling in cancer. J. Recept. Signal. Transduct. Res. 32, 190–195 (2012).2273798010.3109/10799893.2012.695798PMC3503241

[b62] ThieryJ. P. & SleemanJ. P. Complex networks orchestrate epithelial-mesenchymal transitions. Nat. Rev. Mol. Cell Biol. 7, 131–142 (2006).1649341810.1038/nrm1835

[b63] KrishnaS. M., KattoorJ. & BalaramP. Down regulation of adhesion protein E-cadherin in Epstein-Barr virus infected nasopharyngeal carcinomas. Cancer Biomark. 1, 271–277 (2005).1719205110.3233/cbm-2005-1602

[b64] LiuS. J. *et al.* Downregulated NM23-H1 expression is associated with intracranial invasion of nasopharyngeal carcinoma. Br. J. Cancer 98, 363–369 (2008).1821929010.1038/sj.bjc.6604167PMC2361469

The article "Epstein–Barr virus-encoded microRNA BART1 induces tumour metastasis by regulating PTEN-dependent pathways in nasopharyngeal carcinoma" was retracted in 2025. Reasons: contaminated cell lines or tissues; duplicated images; overlap with earlier publications; unreliable data.

[b65] SpruckC. H.3rd *et al.* Absence of p53 gene mutations in primary nasopharyngeal carcinomas. Cancer Res. 52, 4787–4790 (1992).1511442

[b66] WangS. *et al.* RN181 suppresses hepatocellular carcinoma growth by inhibition of the ERK/MAPK pathway. Hepatology 53, 1932–1942 (2011).2139122510.1002/hep.24291

